RETRACTED

# ADAM8 Activates NLRP3 Inflammasome to Promote Cerebral Ischemia-Reperfusion Injury

**DOI:** 10.1155/2021/3097432

**Published:** 2021-12-16

**Authors:** Hongwei Lu, Yaqin Meng, Xinrui Han, Wei Zhang

**Affiliations:** ^1^Key Laboratory for Biotechnology on Medicinal Plants of Jiangsu Province, School of Life Sciences, Jiangsu Normal University, 101 Shanghai Road, Xuzhou 221116, Jiangsu, China; ^2^College of Health Sciences, Jiangsu Normal University, 101 Shanghai Road, Xuzhou 221116, Jiangsu, China

## Abstract

Stroke is the leading cause of death and disability in humans. Strokes are classified as either ischemic or hemorrhagic. Ischemic stroke accounts for 70–80% of the cases. Inflammation is a key factor in ischemic brain injury. Studies have shown that inflammatory response induced by NLRP3 inflammasome is one of the root causes of brain damage in mice with cerebral ischemia. However, its specific mechanism in cerebral ischemia is still unclear. ADAM8 (a disintegrin and metalloproteases 8) is a transmembrane protein with different functions. It plays an important role in tumors and neuroinflammation-related diseases. However, the role and molecular mechanism of ADAM8 in cerebral ischemia injury are still unclear. This study aims to evaluate the role of ADAM8 in cerebral ischemic injury and explore its signal transduction mechanism. This experiment shows that ADAM8 can significantly cause neurological deficits in MCAO mice and can substantially cause ipsilateral cerebral edema and cerebral infarction in MCAO mice. In addition, ADAM8 can significantly induce cortical cell apoptosis in MCAO mice, leading to the loss of neurons and the expression of proinflammatory factors COX2, iNOS, TNF*α*, and IL-6. Importantly, we confirmed that ADAM8 mediates the inflammatory response by promoting the activation of NLRP3 inflammasome, microglia, and astrocytes. These results indicate that ADAM8 may be a candidate drug target for the prevention and treatment of the cerebral ischemic injury.

## 1. Introduction

Stroke can cause disability and death of patients, and it has become one of the public safety issues affecting human health around the world, and ischemic stroke accounts for more than 71% of the cases[1]. In the 1970s, it was discovered that the initial clinical manifestations of stroke patients were mainly hypoperfusion of blood in the penumbra of cerebral ischemia and defects in physiological electrical function. Over time, this area gradually transforms into irreversibly damaged tissue (called the ischemic core), but its transformation rate varies from person to person [2]. Rapid blood flow reperfusion can save brain tissue in the ischemic penumbra and restore normal brain function [3]. This landmark discovery formed the basic principle of reperfusion therapy. Current stroke treatment methods are mainly intravenous thrombolysis and rapid reperfusion of intravascular thrombus removal within 4.5 hours after stroke. Both methods can reduce the risk of death and disability. However, after thrombus removal, thrombolysis, or unexplained thrombosis, the restored blood supply will cause secondary damage. What is more frightening is that this is an irreversible injury, usually accompanied by large areas of cerebral edema, cerebral infarction, or hemorrhagic transformation, which eventually leads to neurological deficits and impaired consciousness, mostly manifested as necrosis of nerve cells in the core area of cerebral infarction [4]. Therefore, there is a dire need to find a broader and safer treatment and it is necessary to establish other treatment strategies.

RETRACTED

Inflammation is an important pathological process of brain injury after cerebral ischemia-reperfusion injury [5]. Inflammatory response begins in the acute phase of stroke and may become the main cause within several hours [6]. The inflammatory response plays an important role in brain injury, and it is a complicated cascading pathological process. It directly destroys the brain tissue structure and affects the blood supply to the injured area. In this process, microglia play an important role [7]. They can secrete inflammation-related cytokines, such as TNF*α*, IL-1*β*, IL-18, and IL-6, and further rise the level of iNOS and MHC class II molecules, destroy the integrity of the blood-brain barrier, and eventually expand infarct and edema volume [8]. Existing studies have shown that the anti-inflammatory factor IL-10 also plays an important role in inflammatory response after cerebral ischemia-reperfusion injury. IL-10 can promote the polarization of microglia into resting-state M2-type microglia and hinder the progress of inflammatory response [9]. However, the exact molecular mechanism of upstream cytokine release is still unclear, which greatly affects clinical treatment.

The innate immunity is closely related to inflammatory processes and predominate in various viral and bacterial infections [10]. At present, researchers have discovered multiple inflammasomes, such as NLRP1, NLRP6, NLRC4, and AIM2 [11]. Among them, NLRP3 inflammasome has been studied most thoroughly. The activated NLRP3 inflammasome can cleave and activate inflammation-related cytokines, such as IL-1*β* and IL-18 [12]. Under certain conditions, caspase-1 can lyse a protein called gasdermin D in the cell, thereby causing cell pyrolysis [13]. At present, studies have confirmed that NLRP3 inflammasome predominates in neuronal cell death and behavioral defects after stroke. Inhibition of NLRP3 inflammasome can protect brain cells from ischemic damage [14]. It indicates the potential therapeutic effect of NLRP3 inflammasome in diseases such as ischemic stroke. There is sufficient evidence that NLRP3 inflammasome plays an important role in the occurrence and development of various major human diseases (such as ischemic stroke and Parkinson's disease). Still, effective clinical drugs that target the NLRP3 inflammasome have not been discovered yet. Therefore, it is particularly important to find the upstream regulatory mechanism of NLRP3 and develop its targeted drugs.

RETRACTED

ADAM8 is highly expressed in diseases characterized by inflammation and tissue remodeling, such as rheumatoid arthritis and asthma [15]. ADAM8 can be induced by inflammatory stimuli such as Lipopolysaccharide (LPS), Interferon-*γ* (IFN-*γ*), and TNF*α*, which further supports its important role in regulating inflammation [16]. At present, there are a few studies about the function of ADAM8 in the nervous system, but all existing studies show that ADAM8 plays a pivotal role in regulating neuroinflammation. Studies have revealed that, in the brain of normal adult mice, ADAM8 expression is low. However, in the mouse model of neurodegeneration, the expression of TNF*α* and ADAM8 both increased significantly [17]. In addition, ADAM8 is also involved in the formation of neural development, myelination, and plasticity proteins, indicating that ADAM8 occupies a central role in the brain and regulation of neuroinflammation. Therefore, it is still necessary to determine the position of ADAM8 in cerebral ischemic injury and its specific molecular mechanism in cerebral ischemic injury.

## 2. Materials and Methods

### 2.1. Animals

120 5-week-old male C57BL/6J mice were purchased from Peng-Yue Experimental Animal Breeding Co., Ltd. Under the conditions of SPF level, Mice had free access to rodent food and tap water under controlled temperature (between 22°C and 24°C) and suitable humidity (60%). Mice were kept on a 12 h light and 12 h dark cycle. After we purchased the mice, we adapted them for a week and then carried out relevant experiments. All mouse experiments complied with Chinese legislation on the use and care of laboratory animals and were approved by the university committees for animal experiments.

### 2.2. Injection of Recombinant Adeno-Associated Virus (AAV)

pAAV-U6-shRNA- (ADAM8-) CMV-EGFP-WPRE-spolyA containing ADAM8 or negative control were purchased from OBiO Technology (Shanghai) Corp., Ltd. The ADAM8 shRNA target sequence is as follows:5′-CCAATGTTCCAGATGTCAA-3′. Injections of either ADAM8 pAAV or control pAAV into the M1 area of the cortex were made at three points relative to bregma (mm): mediolateral axis (ML): ±2 mm, anteroposterior axis (AP): −1 mm, and dorsoventral axis (DV): −1 mm from dura mater at five weeks. Four weeks after surgery, mice were allocated to either Sham or MCAO randomly. The pAAV was injected into cerebral cortex of mice in accordance with the relevant pAAV dose recommended by the company.

RETRACTED

### 2.3. Animal Model

The MCAO/reperfusion is used to establish an ischemic stroke model. The mice were anesthetized with the administration of isoflurane (2% induction, 1.5% maintenance, in 20% oxygen). Body temperature was maintained at 37.0 ± 0.5°C. A silicon-coated monofilament (Jialing, Guangzhou, China) was placed in the internal carotid artery to induce MCAO, and then the monofilament further blocked the middle cerebral artery. The filament was removed for reperfusion after 1 hour. Laser speckle imaging technology (MoorFLPI-2 V2.0, England) was used to confirm MCAO model. We define a successful MCAO model as the cerebral blood flow during ischemia is 75% lower than before. According to the above criteria, the success rate of MCAO mice is 90% of all experimental animals. The Sham operation group was treated with cervical surgery without inserting monofilament. Then the surgical incision was closed, and all the mice returned to their home cages after the operation to get free water and food for recovery.

### 2.4. Neurological Deficit Score

Longa methods [18] were used to assess the neurobehavior of MCAO mice.

0 = no observable deficit; 1 = forelimb flexion; 2 = spontaneous circling to the right; 3 = unilateral circling; 4 = absent ambulation. Therefore, the higher the score, the more severe the neurological dysfunction. Subsequent experiments used MCAO mice with neuron deficiency scores of 1–3.

### 2.5. Infarct Volume and Edema Volume

The brain was taken after reperfusion of 24 hours after the ischemic injury. Subsequently, 2% 2,3,5-triphenyte-trazoliumchloride (Sigma, Missouri, USA) staining was used to assess the infarct volume of 1 mm thick brain slices at 37°C for 10 min. Some photos were taken with a digital camera (Nikon, Tokyo, Japan). ImageJ software was used to evaluate the infarct area of each slice. The percentage of cerebral infarction volume = (cerebral infarct volume/whole brain volume) × 100. We also calculated the rate of edema volume: (ipsilateral hemisphere volume-contralateral hemisphere volume)/whole brain volume × 100 [19].

### 2.6. Brain Slices Collection

The mice were perfused transcardially with normal saline. After incubation overnight at 4°C in PBS containing 30% sucrose, brain tissues were fixed with 4% paraformaldehyde (pH 7.4). Then, the brain tissue was embedded in O.C.T compound (Sakura, Japan). Coronal sections (10 *μ*m) from olfactory bulb tissue were collected.

RETRACTED

### 2.7. Nissl Staining

The Nissl body of neurons was detected by 0.1% Cresyl violet acetate (Sigma, Missouri, USA) staining. The Nissl body of the ipsilateral cortex was measured with ImageJ software.

### 2.8. Terminal Deoxynucleotidyl Transferase-Mediated dUTP Nick-End Labelling Assay (TUNEL)

TUNEL kits (Promega, Madison, USA) were applied to determine the apoptotic cell. Leica Laser Confocal Microscope (Leica, Germany) was used to observe and photograph. TUNEL-positive nuclei stained in green and cells stained with DAPI in blue were counted in random areas. Apoptosis index is expressed as the proportion of apoptosis-positive cells in the nucleus × 100%.

### 2.9. Quantitative Real-Time Polymerase Chain Reaction (RT-qPCR)

Total RNA was extracted by using TRIzol Reagent (Invitrogen, Massachusetts, USA), following the manufacturer's instructions, and then complementary DNA was synthesized with HiScript II qRT SuperMix for qPCR Kit (Vazyme, Nanjing, China). Quantification of ADAM8 level was performed by using the AceQ® qPCR SYBR® Green Master Mix (Vazyme, Nanjing, China) on an ABI StepOnePlus RT-PCR system (Applied Biosystems, Massachusetts, USA) and it was normalized using 2^−△△CT^ method.

### 2.10. Immunoprecipitation Assay

Equal amounts of proteins (1 mg) were precleared with protein A + G-Sepharose beads for 1 hour at 4°C and were then incubated with 2 mg rabbit anti-ADAM8 antibodies (Abbexa, Cambridge, UK) and anti-ADAM8 antibodies (Cell Signaling Technology, Massachusetts, USA) overnight at 4°C. Immune complexes were precipitated using protein A + G-Sepharose beads and were washed four times with 100 mM sodium phosphate buffer (pH 7.4). Following boiling in SDS/PAGE loading buffer, proteins were analyzed by western blot with rabbit anti-ADAM8 (Proteintech, Illinois, USA) and rabbit anti-NLRP3 antibodies (Cell Signaling Technology, Massachusetts, USA).

### 2.11. Western Blot Analysis

Protein was isolated from brain tissues using T-PER™ Tissue Protein Extraction Reagent (Thermo Fisher Scientific, Massachusetts, USA) supplemented with a protease inhibitor mixture (Roche, Basel, Switzerland) and phosphatase inhibitor mixture (Roche, Basel, Switzerland). Equal amounts of total proteins (50 *μ*g) were separated for SDS-PAGE; gels were transferred onto a PVDF membrane (Millipore, Massachusetts, USA). 5% skimmed milk (wt/vol) in Tris-buffered saline containing 0.1% Tween 20 (TBST) was used to incubate membrane for 1 hour at room temperature, and then the membranes were incubated with the corresponding primary antibodies overnight at 4°C. The primary antibodies were as follows: rabbit anti-ADAM8 (1 : 1000; Proteintech, Illinois, USA); rabbit anti-NLRP3 (1 : 1000; Cell Signaling Technology, Massachusetts, USA); mouse anti-iNOS (1 : 1000; Abcam, Cambridge, England); rabbit anti-ASC (1 : 1000; Santa Cruz, California, USA); rabbit anti-Cox2 (1 : 1000; Abcam, Cambridge, England); rabbit anti-caspase1 p20 (1 : 1000; Wanlei, Shenyang, China); mouse anti-TNF*α* (1 : 1000; Abcam, Cambridge, England); rabbit anti-cleaved-IL-1*β* (1 : 1000; Abcam, Cambridge, England); rabbit anti-GFAP (1 : 1000; Abcam, Cambridge, England); and mouse anti-*β*-actin (1 : 1000; AmyJet, China, Wuhan). The blots were incubated with the goat anti-rabbit or anti-mouse HRP-conjugated secondary antibodies (1 : 10000; Millipore, Massachusetts, USA) at room temperature for 1 hour. The chemiluminescence intensity was captured using an AI600 apparatus (GE Healthcare Life Sciences, Uppsala, Sweden) and measured using the ImageJ software.

RETRACTED

### 2.12. Immunofluorescence Staining

The slides were incubated in a 37°C incubator for 120 minutes, and then the slides were recovered for 10 minutes by the sodium citrate antigen recovery method. 5% BSA were added in PBS for 1 hour at room temperature. Then the slides were incubated with primary antibodies overnight at 4°C. The primary antibodies were as follows: rabbit anti-ADAM8(1 : 100; Abbexa, Cambridge, UK); goat anti-NLRP3 (1 : 100; Abcam, Cambridge, UK); chicken anti-GFAP (1 : 500; Abcam, Cambridge, UK); goat anti-Iba-1 (1 : 100; Abcam, Cambridge, UK); and rabbit anti-NeuN (1 : 500, Abcam, Cambridge, UK). On the second day, the slides were rinsed with PBS and incubated with a fluorescent secondary antibody for 1 hour at room temperature. Then, Leica Confocal Laser Microscope was used to capture images and ImageJ software was used to count positive signals and analyze them.

### 2.13. Statistical Analysis

Statistical analysis was done with SPSS software, version 21.0. The data were analyzed with one-way ANOVA followed by Tukey's Honestly Significant Difference post hoc test. Data are expressed as mean ± SD. Statistical significance was set to *P* < 0.05.

## 3. Results

### 3.1. Increased Expression of ADAM8 in the Cerebral Cortex of Mice with Cerebral Ischemia-Reperfusion Injury

Related research in neurodegenerative diseases demonstrates that ADAM8 plays an indispensable role in neuroinflammation [8]. In ischemic stroke, only previous RNA-Seq results of Xu et al. [20] showed that the mRNA level of ADAM8 abnormally increased after one day of cerebral ischemia and reperfusion in mice. Still, there are no other related subsequent studies. Our RT-qPCR study showed that the mRNA level of ADAM8 gradually increased after cerebral ischemia-reperfusion injury of 4 hours, 24 hours, and 72 hours in mice and reached a peak at 72 hours (Figure 1(a)). In addition, the expression level of ADAM8 protein in mice was analyzed by western blot. The results highlighted that there was no significant difference at 4 hours. The protein expression gradually increased after 4 hours, and the expression was at its highest at 72 hours (Figure 1(b)). These results indicate that the expression of ADAM8 is abnormal in mice with cerebral ischemia-reperfusion injury, which may play an unknown functional role. The optimal treatment time is within 4 hours after stroke, after which irreversible damage will occur, and the inflammatory response gradually worsens from 4 hours to 3 days after stroke. Due to the greater damage to the brain caused by MCAO, the mortality rate of the mice was higher after 3 days. Therefore, we selected the study subjects at 24-hour time point after ischemia-reperfusion injury.

RETRACTED

### 3.2. Construction of ADAM8 Knockdown Mouse Model

Gene knockdown or gene silencing is a typical reverse genetics technique, which is often a conventional method for studying the function of a target gene or target protein. RNAi is a small-molecule RNA interference technology discovered in recent years that can specifically recognize, inhibit, and degrade specific mRNA to reduce the expression level of target gene protein without changing DNA. It has been used to silence the target gene to study its role in specific biological activities [21].

The adeno-associated virus was injected into the M1 area of the mouse brain through stereotactic brain technology. Targeted injection of pAAV into M1 region of cerebral cortex not only can make the pAAV fully spread, but also the ischemic penumbra is located in M1 region. After 28 days, the spread of the adeno-associated virus in the mouse cerebral cortex can be observed (Figure 2(a)). Under a 10x magnification microscope, pAAV with EGFP label in M1 area is sufficiently diffused, the adeno-associated virus successfully infects mice cerebral cortex area (Figure 2(b)). Compared with Sham Scramble shRNA mice, the expression of ADAM8 significantly increased in the cortex of MCAO Scramble shRNA mice. After stereotactic injection of ADAM8 shRNA in the brain, the expression of ADAM8 reduced considerably in the cortex of MCAO mice (Figures 2(c) and 2(d)). Our experimental results show that the ADAM8 gene knockdown mouse model was successfully constructed. Our main research object is cerebral cortex in mice; therefore, we will focus on the detection of some cortex-related indicators.

RETRACTED

### 3.3. ADAM8 Induced Cerebral Cortex Injury in Mice with Cerebral Ischemia and Reperfusion

Here, we investigated the role of ADAM8 in brain injury. Longa methods [18] were employed to assess neurological deficits in mice. Mice with cerebral ischemia and reperfusion have obvious defects in nerve function, and knocking down ADAM8 can effectively reverse this situation (Figure 3(a)). Cerebral ischemia-reperfusion mice have larger brain tissue edema and infarct volume on the ischemic side. After knocking down ADAM8, the infarct and edema volume of cerebral ischemia-reperfusion mice was greatly improved (Figure 3(b)). Laser speckle blood flow analysis and Nissl staining are one of the important methods for evaluating cerebral ischemia-reperfusion injury; after knocking down ADAM8 in cerebral ischemia-reperfusion mouse cerebral cortex, it can significantly improve the cerebral blood flow and the loss of Nissl body in cerebral ischemia-reperfusion mice (Figures 3(c) and 3(d)). Our many experimental results have shown that the brain tissue damage of cerebral ischemia-reperfusion mice is extremely serious, which has affected the normal life and physiological activities of mice. After knocking down ADAM8, the brain injury was significantly improved. Therefore, ADAM8 is involved in the pathological process of brain tissue injury in cerebral ischemia-reperfusion mice. However, its specific participation mechanism is currently unclear.

### 3.4. ADAM8 Promotes Neuronal Apoptosis in the Cerebral Cortex of Mice with Cerebral Ischemia-Reperfusion Injury

Apoptosis is the main way of cell death within a few hours after ischemic stroke, and cell apoptosis in the ischemic penumbra can be rescued. Inhibiting cell apoptosis is also an important neuroprotective strategy for ischemic stroke treatment. Protein of cleaved caspase-3 is an executive protein for apoptosis. Our experimental results illustrate that cleaved caspase-3 significantly increased in ischemic penumbra of cerebral cortex. After knocking down ADAM8, the expression of cleaved caspase-3 was inhibited considerably (Figure 4(a)).

To further confirm our findings, in cerebral ischemia-reperfusion mice, we used the TUNEL method to detect apoptosis. It is found that, after knocking down ADAM8, the apoptosis of cerebral ischemia-reperfusion mice cortical neurons was significantly improved (Figure 4(b)). This is consistent with our western blot results.

In summary, after knocking down ADAM8 in cerebral ischemia-reperfusion mice cerebral cortex, it can significantly improve apoptosis in the ischemic penumbra of cerebral ischemia-reperfusion mice.

### 3.5. ADAM8 Promotes Activation of Neuroinflammation in the Cerebral Cortex of Mice with Cerebral Ischemia-Reperfusion Injury

A further study investigates whether ADAM8 participates in the occurrence of cerebral ischemia-reperfusion injury by regulating inflammatory response. The obtained results showed that ADAM8 can promote the expression of some inflammatory factors (iNOS, COX-2, TNF*α*, and IL-6), and neuroinflammatory marker protein GFAP in cerebral ischemia-reperfusion mice. It was observed that ADAM8 can also mediate neuroinflammation by inhibiting the level of anti-inflammatory factor IL-10 in cerebral cortex of mice with cerebral ischemia-reperfusion injury (Figure 5(a)). In addition, generally speaking, there is no inflammatory reaction in neuron cells, so we did not detect the expression of ADAM8 in neuron cells. ADAM8 can promote the activation of astrocytes and microglia, and ADAM8 is expressed in microglia instead of astrocytes (Figures 5(b) and 5(c)).

RETRACTED

### 3.6. ADAM8 Promotes the Activation of NLRP3 Inflammasomes in the Cerebral Cortex of Mice with Cerebral Ischemia and Reperfusion

NLRP3 is the first and most common inflammasome studied in the brain, mainly located in microglia. Its function and binding components have been checked in various brain-related diseases, including ischemic stroke and traumatic brain injury (TBI). From our results, it was concluded that ADAM8 can promote inflammation by activating NLRP3 inflammasomes in mice with cerebral ischemia-reperfusion (Figure 6(a)). To explore the relationship between ADAM8 and NLRP3, our coimmunoprecipitation experiments showed that ADAM8 interacts with NLRP3 (Figure 6(b)). Immunofluorescence further revealed that there is a colocalization between ADAM8 and NLRP3 (Figure 6(c)). These results indicate that there is an interaction between ADAM8 and NLRP3. In summary, ADAM8 may interact with NLRP3 and further activate the NLRP3 inflammasome, promote the occurrence of inflammation, and lead to cerebral ischemia-reperfusion injury ultimately.

## 4. Discussion

Ischemic stroke is a type of cerebral ischemia caused by the reduced blood flow which further induces acute focal brain damage and ultimately leads to neurological deficits [22]. In clinical treatment, t-PA is an effective treatment method for ischemic stroke. However, t-PA also has its time limit and may cause more severe ischemia-reperfusion injury [23]. The inflammatory response after cerebral ischemia-reperfusion injury is a complex cascading pathological process, which not only directly destroys the brain tissue, but also affects the blood supply to the injured site, but it is also one of the main targets for the development of new stroke treatments [8].

RETRACTED

In this study, ADAM8 was expressed in microglia rather than astrocytes. Stroke induced overexpression of ADAM8 in microglia and continued to be expressed and increased within 72 hours. ADAM8 can interact with NLRP3 and activate NLRP3 inflammasomes, mediate the release of IL-1*β* and other proinflammatory cytokines, promote the activation of microglia and astrocytes, stimulate neuroinflammatory responses, and ultimately lead to brain damage. Furthermore, knocking down ADAM8 in the M1 area of the cortex can significantly promote the massive recovery of damaged brain tissue after stroke.

ADAM8 occupies an essential position in promoting the occurrence of inflammatory diseases [15]. In conditions such as tracheal inflammation and rheumatoid arthritis, ADAM8 can encourage the production of many inflammatory factors and ultimately cause tissue damage [24]. In neuroinflammation, ADAM8 can cleave TNF*α* to mediate inflammation [25]. Previously, only RNA-Seq results of Xu et al. [20] showed that, after 24 hours of cerebral ischemia-reperfusion injury, the level of ADAM8 in the ischemic penumbra abnormally increased in ischemic penumbra. However, there is no further report on the function of ADAM8 in cerebral ischemia-reperfusion injury. Therefore, it is speculated that, after cerebral ischemia-reperfusion injury, the level of ADAM8 abnormally increased and leaded to brain damage. The present research validates the previous facts. After cerebral ischemia-reperfusion injury, the level of ADAM8 in microglia increased rapidly, resulting in defects to neurological function of mice with cerebral ischemia-reperfusion injury. Infarcts and edema of brain, insufficient blood supply to the brain, and loss of brain neurons eventually caused brain damage in mice with cerebral ischemia-reperfusion injury.

Inflammation is an important reason of brain injury after cerebral ischemia-reperfusion injury [8]. DAMP-related molecules are released rapidly after cerebral ischemia-reperfusion injury occurs. And these DAMP-related molecules trigger sterile inflammatory response. In this process, the first responding immune cell is the microglia [26]. Once activated, microglia release molecules that further recruit neutrophils, monocytes, and lymphocytes [27]. In addition, cerebral ischemia-reperfusion injury will trigger complement system, which further mediates the expansion of the inflammatory response [28]. Activated microglia can also activate astrocytes by secreting Il-1*α*, C1q, and TNF. After astrocytes are activated, they can also secrete a neurotoxin, leading to the rapid death of other nerve cells, such as neurons and oligodendrocytes. Activated astrocytes will upregulate many classic complement system related genes, which have been shown to trigger neuroinflammation further and have destructive effects on nerve synapses. After the activation of astrocytes was inhibited, the death of neurons was significantly improved [29]. Previous studies reported that, in diseases such as tracheal inflammation and rheumatoid arthritis, ADAM8 can activate NF-*κ*B, JNK, p38, and other inflammation-related signal pathways, thereby producing inflammatory factors and amplifying the inflammatory cascade, eventually causing tissue damage [24]. In neuroinflammation such as Parkinson's and Alzheimer's disease, there are also reports that ADAM8 plays a pivotal role in promoting the release of inflammatory factors such as TNF*α* [17]. Therefore, it is speculated that ADAM8 abnormally increased, and it caused brain damage by stimulating neuroinflammatory responses after cerebral ischemia-reperfusion injury. The present research also substantiates this point. After cerebral ischemia-reperfusion injury, the level of ADAM8 in microglia rises rapidly, which promotes the release of a series of inflammatory factors (iNOS, COX2, TNF*α*, IL-1*β*, and IL-6) and inhibits the level of anti-inflammatory factor IL-10. It further activates microglia and astrocytes and severely damages the brain tissue after ischemia and reperfusion.

RETRACTED

The activated NLRP3 inflammasome can induce inflammatory response in many types of diseases. NLRP3 inflammasome predominates in inflammatory response. Targeted inhibition of NLRP3 inflammasome has a significant preventive or therapeutic effect [30]. Studies have confirmed that NLRP3 inflammasome had a leading role in neuronal cell death and behavioral defects after stroke, and inhibition of NLRP3 inflammasome can protect brain cells from ischemic damage [14]. It indicates the potential therapeutic effects of NLRP3 inflammasome in brain-related diseases such as ischemic stroke. However, there are few effective clinical drugs that target the inhibition of NLRP3 inflammasomes. Therefore, it is particularly important to find the upstream regulatory mechanism of NLRP3 and develop related new drugs. At present, published studies preach that, after cerebral ischemia-reperfusion injury, NLRP3 can boost the level of inflammatory factors through the NLRP3/NF-*κ*B axis. As the most comprehensively studied inflammasome in the brain, it is not difficult to speculate that ADAM8 may be related to the NLRP3 inflammasome, thereby activating the NLRP3/NF-*κ*B axis and mediating the occurrence of inflammation. Holistic investigation showed that ADAM8 can interact with NLRP3, further activate the NLRP3 inflammasome, and cause the occurrence of inflammation. In a nutshell, we preliminarily verified the correlation between ADAM8 and NLRP3, but it is not clear whether it has direct interaction or indirect interaction, which will be further discussed in our follow-up study.

RETRACTED

## 5. Conclusion

In conclusion, this study reveals possible molecular mechanism of ADAM8-mediated cerebral ischemia-reperfusion injury. For the first time, we found that the expression of ADAM8 is abnormally increased, and it eventually leads to brain damage after ischemia-reperfusion injury by promoting the activation of NLRP3 inflammasome. Neurological deficit score was used to evaluate the neurological function of cerebral ischemia-reperfusion mice and TTC staining and laser blood flow speckle imaging were made to measure the mice' cerebral cortex damage. Nissl staining and TUNEL were used to explore the neuron loss in brain injury. In addition, immunofluorescence was used to detect the microglia activation and NLRP3 followed by western blots to identify the expression of the NLRP3/NF-*κ*B axis and neuroinflammation-related proteins. We also preliminarily explained the connection between ADAM8 and NLRP3 through coimmunoprecipitation. We found that ADAM8 can induce neuroinflammation and cause cerebral ischemia-reperfusion injury by mediating NLRP3 inflammasome activation, and knocking down ADAM8 can greatly alleviate cerebral ischemia-reperfusion injury. All in all, after cerebral ischemia-reperfusion injury, the level of ADAM8 rises rapidly. ADAM8 further activates NLRP3 inflammasome by interacting with NLRP3, mediates inflammatory response, promotes the release of inflammatory factors, and eventually causes brain tissue damage. Specific knock down of ADAM8 can significantly alleviate cerebral ischemia-reperfusion injury. The proposed study provides a new mechanism of cerebral ischemia-reperfusion injury and offers new ideas for the treatment strategy after cerebral ischemia-reperfusion injury.

## Figures and Tables

**Figure 1:** Expression of ADAM8 in cerebral cortex of ischemia-reperfusion mice increased abnormally. (a) QPCR analysis of ADAM8 levels in mouse cerebral cortex, *n* = 3 mice per group. (b) Brain homogenates of the indicated group were obtained after reperfusion for 4/24/72 hours. And the level of the indicated proteins was analyzed with western blotting, *n* = 4 mice per group. All values are expressed as the mean ± SD. ^*∗*^*P* < 0.05, ^*∗∗*^*P* < 0.01, ^*∗∗∗*^*P* < 0.001 vs. Sham group. ^#^*P* < 0.05, ^##^*P* < 0.01, ^###^*P* < 0.001 vs. MCAO group.

**Figure 2:** Strategy for generating the ADAM8 gene knockdown mice. (a) Effect of stereotactic cerebral injection, *n* = 4 mice per group. (b) Immunofluorescence analysis of adeno-associated virus in primary motor cortex region of mice 28 days after injection. Adeno-associated viruses carry green fluorescent protein (EGFP) and DAPI (blue) stains the nucleus (scale = 200 *μ*m). The magnification is 10x, *n* = 3 mice per group. (c) After reperfusion for 24 hours, the effects of different shRNA fragments were analyzed with western blotting, *n* = 5 mice per group. (d) The expression of ADAM8 in the cortex of mice in different treatment groups was detected by immunofluorescence staining, the magnification is 40x, and the scale bar was 50 *μ*m, *n* = 5 mice per group. All values are expressed as the mean ± SD. ^*∗*^*P* < 0.05, ^*∗∗*^*P* < 0.01, ^*∗∗∗*^*P* < 0.001 vs. Sham Scramble shRNA group. ^#^*P* < 0.05, ^##^*P* < 0.01, ^###^*P* < 0.001 vs. MCAO Scramble shRNA group.

RETRACTED

**Figure 3:** ADAM8 induced cerebral cortex injury induced in cerebral ischemia-reperfusion mice. (a) After reperfusion for 24 hours, neurological deficits of mice were assessed, *n* = 8 mice per group. (b) After reperfusion for 24 hours, brain sections of the indicated group were stained with 2,3,5-triphenyltetrazolium chloride (left) and analysis of infarct volume (right) was performed, *n* = 5 mice per group. (c) After reperfusion for 24 hours, cerebral blood flow of mice was recorded, *n* = 4 mice per group. (d) Nissl staining assays were performed in ischemic brain sections at 24 hours after I-R injury, *n* = 4 mice per group. All values are expressed as the mean ± SD. ^*∗*^*P* < 0.05, ^*∗∗*^*P* < 0.01, ^*∗∗∗*^*P* < 0.001 vs. Sham Scramble shRNA group. ^#^*P* < 0.05, ^##^*P* < 0.01, ^###^*P* < 0.001 vs. MCAO Scramble shRNA group.

**Figure 4:** ADAM8 promoted the apoptosis of cerebral cortical neurons in cerebral ischemia and reperfusion mice. (a) Cleaved caspase-3 in the penumbra was detected by western blotting after reperfusion for 24 hours, *n* = 4 mice per group. (b) TUNEL and immunofluorescence analysis of the apoptosis cerebral in cortex penumbra at 24 hours after I-R injury. The magnification was 40x and the scale bar was 50 *μ*m, *n* = 3 mice per group. All values are expressed as the mean ± SD. ^*∗*^*P* < 0.05, ^*∗∗*^*P* < 0.01, ^*∗∗∗*^*P* < 0.001 vs. Sham Scramble shRNA group. ^#^*P* < 0.05, ^##^*P* < 0.01, ^###^*P* < 0.001 vs. MCAO Scramble shRNA group.

**Figure 5:** ADAM8 promoted neuroinflammation in cerebral ischemia-reperfusion mice. (a) Western blot analysis of proteins was associated with inflammation after reperfusion for 24 hours, *n* = 3 mice per group. (b) and (c) immunofluorescence analysis of GFAP and Iba-1 in cortex penumbra at 24 hours after I-R. The magnification was 40x and the scale bar was 50 *μ*m, *n* = 3 mice per group. All values are expressed as the mean ± SD. ^*∗*^*P* < 0.05, ^*∗∗*^*P* < 0.01, ^*∗∗∗*^*P* < 0.001 vs. Sham Scramble shRNA group. ^#^*P* < 0.05, ^##^*P* < 0.01, ^###^*P* < 0.001 vs. MCAO Scramble shRNA group.

RETRACTED

**Figure 6:** ADAM8 activated NLRP3 inflammasome in cerebral cortex of cerebral ischemia-reperfusion mice. (a) Western blotting reflected the relative level of indicated proteins in different groups after I-R 24 hours, *n* = 3 mice per group. (b) The interaction between ADAM8 and NLRP3 in cerebral cortex of I-R mice, *n* = 3 mice per group. (c) Immunofluorescence analysis of brain sections with antibodies specific for ADAM8 and NLRP3 (colocalization of ADAM8 with NLRP3). The magnification was 40x and the scale bar was 50 *μ*m. All values are expressed as the mean ± SD. ^*∗*^*P* < 0.05, ^*∗∗*^*P* < 0.01, ^*∗∗∗*^*P* < 0.001 vs. Sham Scramble shRNA group. ^#^*P* < 0.05, ^##^*P* < 0.01, ^###^*P* < 0.001 vs. MCAO Scramble shRNA group.

## Data Availability

No data were used to support this study.
